# Clinical Study of Clopidogrel Combined with Huoxue Tongluo Prescription in Improving Transient Ischemic Attack and the Effect on MMP-9, Hcy, and CRP

**DOI:** 10.1155/2022/6368219

**Published:** 2022-03-31

**Authors:** Lifang Ma, Zhe Chen, Yan'e Li, Xin Meng, Yongsheng Ma

**Affiliations:** ^1^Department of Clinical Laboratory, People's Hospital of Rizhao, Rizhao 276800, China; ^2^School Health Supervision Office, Health and Family Planning Inspection Agency of Zhangqiu Dictrict, Jinan 250200, China; ^3^Department of Medicine, Zhangqiu District People's Hospital, Jinan 250200, China; ^4^Department of Traditional Chinese Medicine, Qingdao Eighth People's Hospital, Qingdao 266000, China; ^5^Health Care Department, Weifang People's Hospital, Weifang 261041, China

## Abstract

**Background:**

This study aimed to explore the clinical study of clopidogrel combined with Huoxue Tongluo prescription in improving transient ischemic attack (TIA) and the effect on MMP-9, Hcy, and CRP.

**Methods:**

A total of 84 patients with TIA admitted to our hospital from December 2019 to February 2021 were selected. The patients were divided into the control group (42 cases: not treated with Huoxue Tongluo prescription) and study group (42 cases: treatment with Huoxue Tongluo prescription). The clinical efficacy, adverse reactions, the levels of blood pressure and lipid, blood rheology and cerebral hemodynamics, neurological function-related indicators, MMP-9, Hcy, and CRP of the two groups were compared.

**Results:**

The total effective rate in the study group was higher than the control group. Compared with before treatment, the levels of SBP and DBP in both groups decreased memorably after treatment, and those in the study group decreased more particularly than the control group. The levels of LDL, HDL, TC, and TG in the study group were significantly better than those in the control group. The plasma viscosity, whole blood high shear viscosity, whole blood low shear viscosity, and hematocrit of patients in the study group were lower than those in the control group, and the maximum blood flow velocity, minimum blood flow velocity, average blood flow velocity, and average blood flow were higher than those in the control group. The levels of NSE, MBP, and S100*β* in the study group were more memorably lower than those in the control group. After treatment, the levels of MMP-9, Hcy, and CRP in the study group were significantly lower than those in the control group. There was no obvious difference in the incidence of adverse reactions between the study group and control group.

**Conclusion:**

Clopidogrel combined with Huoxue Tongluo prescription can significantly improve the therapeutic effect and reduce the levels of MMP-9, Hcy, and CRP in patients with TIA.

## 1. Introduction

Transient ischemic attack (TIA) refers to the transient insufficiency of blood supply in the carotid artery and vertebrobasilar artery system, resulting in focal cerebral ischemia. TIA is most common in the elderly and clinically manifested as short-term focal neurological dysfunction. TIA has the characteristics of high incidence and recurrence rate. In general, its attack time usually lasts 10–15 minutes, and the patient can recover within 30 minutes. If the attack time exceeds 2 hours, the neurological function of the patient will be damaged [1, 2]. Patients with cerebrovascular diseases such as hypertension, diabetes, dyslipidemia, atherosclerosis, and heart disease are prone to TIA. Because, the oxidative stress in the cerebrovascular system will cause endothelial dysfunction, which disrupts the balance in blood vessels and leads to TIA. TIA is a high risk factor for stroke. TIA patients can develop severe cerebral infarction and even death if they are not treated promptly and effectively [3]. Therefore, it is of great significance to select reasonable drugs for treatment and improve the safety of treatment after TIA. The pathogenesis of TIA is complex, and currently, thromboembolism, microembolism, and hypoperfusion are considered to be the main pathogenesis. Clopidogrel [4] is a commonly used drug in clinical treatment of cerebral ischemia, which can avoid brain tissue damage to a certain extent. But the remission rate of Western medicine alone is less than 70%, and the recurrence rate is high. According to the etiology and pathogenesis of cerebral ischemia proposed in traditional Chinese medicine, it can be treated with drugs from the perspectives of facilitating blood circulation and removing stasis, tonifying blood, and activating qi. The combination of drugs in Huoxue Tongluo prescription has the effects of promoting blood circulation and removing blood stasis, clearing the heart and opening the body, regulating qi, improving blood lipids and other indicators of patients, and can also alleviate vertigo symptoms of patients during attacks [5].

Therefore, 84 TIA patients were selected for clopidogrel combined with Huoxue Tongluo prescription, aiming to analyze the therapeutic effect and its influence on MMP-9, Hcy, and CRP levels of patients, so as to provide reliable data support for clinical research.

## 2. Materials and Methods

### 2.1. General Data

A total of 84 TIA patients admitted to our hospital from December 2019 to February 2021 were selected as the study subjects. With the consent of the patients, they were divided into the control group (*n* = 42) and study group (*n* = 42) by the random number table method. There were 27 males and 15 females in the control group. The average age was (66.2 ± 5.7) years. There were 24 patients with hypertension and 18 patients with hyperlipidemia. There were 25 males and 17 females in the study group. The average age was (67.4 ± 5.3) years. There were 26 patients with hypertension and 16 patients with hyperlipidemia. There was no obvious difference in general data between the study group and control group (*p* > 0.05). Inclusion criteria: patients who met the relevant diagnostic criteria of TIA [6]; after clinical examination and related imaging examination, all patients were diagnosed with TIA; patients who received treatment; and patients who signed the informed consent forms. Exclusion criteria: patients with the history of cerebral infarction and cerebral hemorrhage; patients with other serious cardiovascular, cerebrovascular, liver, and kidney dysfunction; patients with malignant tumors; patients with missing or incomplete data; and patients allergic to the drugs in this study.

### 2.2. Therapeutic Methods

All patients received routine treatment, including vasodilation, anticoagulation, and control of underlying diseases. The control group was treated with clopidogrel orally (H20120035, Shenzhen Salubris Pharmaceuticals Co., Ltd.), 75 mg/time, once a day. The study group was treated with Huoxue Tongluo prescription [7] on the basis of the control group. Recipe composition: Calculus Bovis Artifactus 0.2 g, leech 3 g, Bile Arisaema 10 g, safflower 10 g, *Angelica* 15 g, peach kernel 15 g, *Ginkgo* leaf 15 g, *Acorus tatarinowii* 15 g, Radix Paeoniae Rubra 15 g, earthworm 20 g, *Ligusticum wallichii* 25 g, and *Astragalus* 30 g. One dose of Huoxue Tongluo prescription was decocted with water to 300 ml every day and taken twice in morning and evening, 150 ml/time. Both groups were treated for 3 months.

### 2.3. Observational Index

#### 2.3.1. The Clinical Efficacy

Healed: transient vertigo, aphasia, monocular visual impairment, and other symptoms were disappeared after treatment, and there was no recurrence in 3 months follow-up. Improved: the above symptoms were significantly improved, and the frequency and duration of the disease were notably reduced, and the recurrence was ≤2 times within 3 months of follow-up. Ineffective: the patient's disease control effect was not good after treatment, with no significant improvement or even aggravation of symptoms, the recurrence was ≥3 times within 3 months of follow-up, and patients have prolonged illness or progress to cerebral infarction [8]. Total effective rate = recovery rate + improvement rate.

#### 2.3.2. Blood Pressure

The blood pressure of the two groups were compared before treatment and 3 months after treatment. The diastolic and systolic blood pressure were measured with a blood pressure monitor carried in the stool, and professionals were arranged to measure the blood pressure.

#### 2.3.3. Blood Lipid Level

The blood lipid levels of the two groups were contrasted before and 3 months after treatment. Reference for normal blood lipid value [9]: TC level is about 3–5.2 mmol/L; TG level is about 1.7 mmol/L; HDL-C >1.04 mmol/L; and LDL-C < 3.12 mmol/L.

#### 2.3.4. Hemorheological Indexes and Hemodynamic Indexes

The hemorheological indexes and hemodynamic indexes of the two groups were compared before treatment and 3 months after treatment. The plasma viscosity, high whole blood viscosity, hematocrit, low whole blood viscosity, maximum blood velocity, minimum blood velocity, average blood flow, and average blood velocity of the patients were recorded.

#### 2.3.5. Neurological Function-Related Indicators

The neurological function indexes of the two groups were compared before and after treatment for 3 months. The contents of S100*β*, NSE, and MBP were determined by ELISA.

#### 2.3.6. MMP-9, Hcy, and CRP Level

MMP-9, Hcy, and CRP levels were compared between the two groups. In morning, fasting venous blood (5 ml) was centrifuged to separate serum. ELISA was performed to test the levels of MMP-9, Hcy, and CRP by the automatic biochemical analyzer (BK-1200, Shandong Boke Biological Industry Co., Ltd., China). The kit was purchased from Abbott (USA).

#### 2.3.7. Adverse Reaction Rate

The rate of adverse reaction during treatment was compared between the two groups. Medical staff regularly observed and recorded the occurrence of adverse reactions. Adverse reactions include subcutaneous mucosal hemorrhage, gastrointestinal reactions, abnormal liver function, abdominal distension, and headache.

### 2.4. Statistical Analysis

SPSS 22.0 software was used to analyze the data. The counting data were expressed as percentage (%) and performed by the *χ*^2^ test. The measurement data were expressed as $\left(\bar{x}\pm s\right)$, the independent sample *t*-test was performed for comparison between the two groups, and the paired *t*-test was performed for comparison within the groups. *P* < 0.05 indicated that the difference was statistically significant.

## 3. Results

### 3.1. The Clinical Efficacy Was Compared between the Two Groups

After treatment, 26 patients in the study group were healed, 14 patients were improved, and 2 patients were ineffective; the total effective rate was 95.24%. In the control group, 17 patients were healed, 16 patients were improved, and 9 patients were ineffective; the total effective rate was 78.57%. There was no remarkable difference in general data between the two groups (*p*=0.039, Table 1).

### 3.2. Blood Pressure Levels Were Compared between the Two Groups

There was no remarkable difference in blood pressure between the two groups before treatment (*p* > 0.05). After treatment, the levels of SBP and DBP in two groups were sharply decreased than those before treatment (*p* < 0.05), and the decrease in the study group was more obvious than the control group (*p* < 0.05, Figure 1).

### 3.3. The Serum Lipid Levels Were Compared between the Two Groups

Before treatment, no notable differences in LDL, HDL, TC, and TG between the study group and control group were discovered (*p* > 0.05). After treatment, the levels of LDL, TC, and TG in two groups were remarkably lower than before (*p* < 0.05), while the HDL level in both groups was higher than before (*p* < 0.05). The levels of LDL, HDL, TC, and TG in the study group were clearly better than those in the control group (*p* < 0.05, Figure 2).

### 3.4. The Hemorheological Indexes and Cerebral Hemodynamic Indexes Were Compared between the Two Groups

Compared with the control group, the plasma viscosity, whole blood high shear viscosity, whole blood low shear viscosity, and hematocrit of patients were lower in the study group after treatment. The study group's average blood flow velocity, maximum blood flow velocity, minimum blood flow velocity, and average blood flow were higher than those in the control group (*p* < 0.05, Table 2).

### 3.5. The Nerve Function Related Indexes between the Two Groups Were Contrasted

There were no notable differences in NSE, MBP, and S100*β* levels between the two groups before receiving treatment (*p* > 0.05). Compared with pretreatment, the levels of NSE, MBP, and S100*β* in the two groups were sharply lower after treatment, and the decrease in the study group was more obvious (*p* < 0.05, Figure 3).

### 3.6. MMP-9, Hcy, and CRP Levels Were Compared between the Two Groups

There were no obvious differences in MMP-9, Hcy, and CRP levels between the two groups before treatment (*p* > 0.05). After treatment, the levels of MMP-9, Hcy, and CRP in the two groups were clearly lower than before treatment (*p* < 0.05). Compared with the control group, MMP-9, Hcy, and CRP were obviously lower in the study group (*p* < 0.05, Figure 4).

### 3.7. The Comparison of Adverse Reactions Rate between the Two Groups

In the study group, subcutaneous mucosal hemorrhage, gastrointestinal reaction, abnormal liver function, abdominal distension, and headache occurred in 1, 5, 1, 4, and 2 cases, respectively. In the control group, subcutaneous mucosal hemorrhage, gastrointestinal reaction, abnormal liver function, abdominal distension, and headache occurred in 2, 4, 2, 5, and 1 cases, respectively (Table 3).

## 4. Discussion

TIA, a common cerebrovascular disease, is a neurological disorder caused by focal and transient cerebral ischemia, and its clinical manifestations are unclear speech expression, transient nystagmus, reduced vision, tinnitus, unstable standing or walking, and vertigo [10]. Modern medical research believes [11–13] that the onset of TIA is related to the formation of carotid atherosclerotic plaque, high cholesterol, and abnormal hemodynamics. The basic pathological changes of TIA are insufficient blood supply to the brain tissue, which can affect the normal function of nerve cells. Meanwhile, brain tissue may undergo necrosis due to hypoxia and ischemia, thus damaging the central nervous function of patients and increasing the risk of cerebral hemorrhage, cerebral infarction, and other serious cerebrovascular diseases. If TIA is not controlled in time, it may lead to hemiplegia, body and language dysfunction, or even threaten the patient's life. Clinically, the key of Western medicine in the treatment of TIA is to reduce cholesterol level, reduce blood viscosity, and inhibit the formation of thrombosis by controlling platelet aggregation [14]. Clopidogrel [15] is the most widely used drug with significant short-term efficacy and good safety and does not increase the occurrence of hemorrhagic stroke and other adverse reactions. According to traditional Chinese medicine [16], cerebral ischemia can be classified into the category of “blood stasis syndrome,” and the pathogenic mechanism is blood stasis block and qi and blood obstruction. Therefore, TIA is treated by supplementing qi and promoting blood circulation and clearing collaterals and meridians.

In this study, the treatment efficiency of the study group was clearly higher than that of the control group. The levels of TG, TC, LDL, SBP, and DBP in the study group were lower, while the HDL level was higher than the control group. This is because Huoxue Tongluo prescription has the effect of removing stasis, promoting qi, dredging collaterals, and opening orifices. Among them, *Astragalus* and *Ligusticum wallichii* can nourish qi, strengthen the spleen, and regulate qi. Earthworm and *Ginkgo* leaf can regulate meridians, activate collaterals, remove turbidity, and reduce lipids, so as to inhibit blood viscosity, fibrinogen content, and other indicators of patients and play a certain role in improving blood lipids and blood pressure of patients [17, 18]. Patients with recurrent cerebral ischemia will have their own neurological function affected. Serum MBP, S100*β*, and NSE are specific indicators of neurological function evaluation, and the levels are positively correlated with the severity of the disease [19, 20]. Recently, cerebral blood flow of patients with TIA is relatively abnormal, mainly manifested as increased resistance, and both cerebral blood flow and velocity have a downward trend. Compared with the control group, the levels of MBP, S100*β*, and NSE in the study group were lower. After treatment, the indexes of cerebral blood flow in both groups were improved, and the study group was better than the control group. These results indicated that Huoxue Tongluo prescription combined with clopidogrel has an ideal repair effect on patients with nerve damage and can also effectively improve the cerebral blood flow status. Safflower is a good medicine for activating blood circulation and removing blood stasis. *Angelica* invigorates blood circulation. *Ligusticum wallichii* can regulate Huoxue Tongmai. *Acorus tatarinowii* can regulate qi Kaiqiao. *Ginkgo* leaf can regulate Tongluo lowering fat. Peach kernel can regulate Tongluo and Huoxue Huayu. Radix Paeoniae Rubra can nourish blood and activate blood and nourish qi and blood. Earthworm can promote blood circulation and remove blood stasis. The whole prescription has the effect of promoting blood circulation and qi circulation, invigorating the body and clearing the mind [21–23]. Reports confirmed [24–26] that *Ginkgo* leaf and *Astragalus* can effectively reduce arterial blood flow velocity, while *Ligusticum wallichii* has the effect of anticoagulation and improving brain circulation. Moreover, there was no increase in adverse reactions after the use of Huoxue Tongluo prescription, indicating its high safety and can be applied to the treatment of patients with TIA.

MMP-9 [27] controls the degradation and remodeling of extracellular matrix and is involved in the formation of atherosclerosis, increasing the risk of plaque rupture. Under normal circumstances, the expression of MMP-9 in brain tissue is at a low level. But when cerebral ischemia occurs, local inflammatory reaction makes MMP-9 greatly expressed in ischemic tissue. MMP-9 expression is more obvious in tissues with more severe ischemia. Vafadari B believed that MMP-9 played a significant role in the pathological process of secondary brain injury after cerebral infarction and may be a new biological indicator for predicting cerebral infarction [28]. Hcy [29] is an important intermediate product in the metabolic pathway of sulfur-containing amino acids such as cysteine and methionine. However, as a sulfur-containing 4-carbon *α*-amino acid, it does not participate in protein synthesis, but participates in the reaction of vascular damage. Elevated Hcy level is closely related to cardiovascular diseases, which can lead to platelet aggregation and induce thrombosis by promoting oxygen free radical generation and damaging vascular endothelial cells. CRP [30], as an acute phase protein in inflammatory response, is significantly higher than normal when the body has serious infection, ischemia, and other changes. Clinical studies have confirmed [31] that changes in the CRP level are helpful to understand the disease progression and occurrence of cerebral infarction in TIA. The higher the serum CRP level, the more likely the patient is to develop a cerebral infarction The results displayed that Huoxue Tongluo prescription effectively downregulated MMP-9, Hcy, and CRP levels. The mechanism may be related to the improvement of cerebral blood circulation and blood supply and antiplatelet aggregation in patients with TIA.

## 5. Conclusion

In conclusion, Huoxue Tongluo prescription combined with clopidogrel can effectively improve the blood lipid and blood pressure levels and cerebral blood flow status of TIA patients, regulate the levels of MMP-9, Hcy, and CRP, and repair damaged nerves, with good safety and significant efficacy.

## Figures and Tables

**Figure 1:** Comparison of blood pressure levels between the two groups. (a) The comparison of SBP levels between the two groups before and after treatment. (b) The comparison of DBP levels between the two groups before and after treatment. ^*∗*^*P* < 0.05, compared with before treatment. ^Δ^*P* < 0.05, compared with the control group.

**Figure 2:** Comparison of blood lipid levels between the two groups. (a) The comparison of LDL levels between the two groups before and after treatment. (b) The comparison of HDL levels between the two groups before and after treatment. (c) The comparison of TC levels between the two groups before and after treatment. (d) The comparison of TG levels between the two groups before and after treatment. ^*∗*^*P* < 0.05, compared with before treatment. ^Δ^*P* < 0.05, compared with the control group.

**Figure 3:** Comparison of neurological function-related indexes between the two groups. (a) The comparison of NSE levels between the two groups before and after treatment. (b) The comparison of MBP levels between the two groups before and after treatment. (c) The comparison of S100*β* levels between the two groups before and after treatment.

**Figure 4:** Comparison of MMP-9, Hcy, and CRP levels between the two groups. (a) The comparison of MMP-9 levels between the two groups before and after treatment. (b) The comparison of Hcy levels between the two groups before and after treatment. (c) The comparison of CRP levels between the two groups before and after treatment.

**Table 1:** Comparison of clinical efficacy between the two groups.

Groups	*n*	Healed	Improved	Ineffective	Total effective rate
Study group	42	26	14	2	40 (95.24%)
Control group	42	17	16	9	33 (78.57%)
*χ* ^2^					6.472
*P*					0.039

**Table 2:** Comparison of hemorheological indexes and cerebral hemodynamic indexes between the two groups after treatment (‾*x* ± *s*).

Indicators		Study group (*n* = 42)	Control group (*n* = 42)	*t*	*P*
Hemorheological index	Plasma viscosity (m Pa·s)	0.38 ± 0.19	2.48 ± 0.60	21.59	<0.001
	Whole blood high shear viscosity (m Pa·s)	1.03 ± 0.17	4.60 ± 0.29	68.84	<0.001
	Whole blood low shear viscosity (m Pa·s)	9.08 ± 0.09	11.07 ± 0.46	27.36	<0.001
	Hematocrit (%)	40.08 ± 1.03	43.85 ± 2.37	9.452	<0.001

Cerebral hemodynamic indexes	Maximum blood flow velocity (cm/s)	43.21 ± 4.65	40.40 ± 4.73	2.748	0.007
	Minimum blood flow velocity (cm/s)	12.26 ± 2.42	9.96 ± 1.78	4.954	<0.001
	Mean blood flow velocity (cm/s)	21.34 ± 3.53	14.64 ± 3.76	8.415	<0.001
	Mean blood flow (m L/s)	11.79 ± 2.33	9.33 ± 1.78	5.436	<0.001

**Table 3:** Comparison of adverse reactions between the two groups (*n*).

Group	*n*	Subcutaneous mucosal hemorrhage	Gastrointestinal reaction	Abnormal liver function	Abdominal distension	Headache
Study group	42	1	5	1	4	2
Control group	42	2	4	2	5	1

## Data Availability

The datasets used and/or analyzed during the current study are available from the corresponding author upon request.
